This article has been retracted.

# Evaluation of Chronic Nanosilver Toxicity to Adult Zebrafish

**DOI:** 10.3389/fphys.2017.01011

**Published:** 2017-12-14

**Authors:** Roberta Pecoraro, Fabio Marino, Antonio Salvaggio, Fabiano Capparucci, Gianfranco Di Caro, Carmelo Iaria, Andrea Salvo, Archimede Rotondo, Daniele Tibullo, Giulia Guerriero, Elena M. Scalisi, Massimo Zimbone, Giuliana Impellizzeri, Maria V. Brundo

**Affiliations:** ^1^Department of Biological, Geological and Environmental Science, University of Catania, Catania, Italy; ^2^Department of Chemical, Biological, Pharmaceutical and Environmental Sciences, University of Messina, Messina, Italy; ^3^Experimental Zooprophylactic Institute of Sicily, Catania, Italy; ^4^Department of Veterinary Sciences, University of Messina, Messina, Italy; ^5^Department of Biomedical, Dental and Morphological and Functional Sciences, University of Messina, Messina, Italy; ^6^Department of Biomedical and Biotecnological Sciences, University of Catania, Catania, Italy; ^7^Department of Biology, University of Naples Federico II, Naples, Italy; ^8^CNR-IMM, Catania, Italy

**Keywords:** *Danio rerio*, AgNPs, inducible metallothioneins, ICP-MS, PLAL

## Abstract

Nanotechnology is rapidly growing with nanoparticles produced and utilized in a wide range of commercial products worldwide. Among the different types of nanomaterials produced, silver nanoparticles (AgNPs) occupy a predominant position and they are used in electronics, clothing, food industry, cosmetics and medical devices. Nanosilver has also showed excellent performance in antibacterial application. Nowadays, the increasing use of AgNPs has put the evidence on their possible toxicity to the human health and the impact on the environment. This paper focus on adverse effects of AgNPs in adult of *Danio rerio*. Fishes exposed to increasing concentrations (8, 45, and 70 μg/l) silver nanoparticles (AgNPs, 25 nm in average diameter) and after treatment for 30 days, was quickly euthanized in MS-222. We have evaluated bioaccumulation of AgNPs using ICP-MS and analyzed histological changes, biomarkers of oxidative damage and gene expression in the gut, liver and gills tissues of AgNPs-treated zebrafish. The histological analysis showed lesions of secondary lamellae of the gills with different degrees of toxicity such as hyperplasia, lamellar fusion, subepithelial edema, and even in some cases telangiectasia. Huge necrosis of the intestinal villi was found in the gut. No lesion was detected in the liver. The analysis revealed a high expression of metallothioneins 1 (MTs 1) in animals exposed to AgNPs compared to the control group. The ICP-MS analysis shows that the amount of particles absorbed in all treated samples is almost the same. We can affirm that AgNPs toxicity linked more to their size and state of aggregation than to their concentrations. Silver nanoparticles can damage gills and gut because they are able to pass through the mucosal barrier thanks to their small size. The damage is still reversible because it is not documented injury to the basal membrane.

## Introduction

In recent decade, nanomaterials (NMs) have attracted much attention because of their many technologically interesting properties. Nanotech applications advance very quickly while very little has been done to measure and assess the risks of nanoparticles in biological systems and ecosystems. There is a strong debate among scientists about the benefits of nanotechnology for humans, but also on the risks to human and environmental health toward several engineered nanomaterials that have become commercial consumer products (Owen and Handy, 2007). It would be appropriate asking some questions about the use of NMs because it raised some concerns: could these substances be more toxic, more mobile, more persistent than their bulk materials? Could they be harmful to environment and human health when manufactured in nanosize? Which are the ways of absorption of nanoparticles and what damage they can cause in fishes?

Studies demonstrate that NPs can be released in the environment and cause harmful effects to all living organisms (Owen and Depledge, 2005; Scuderi et al., 2014). Several *in vivo* and *in vitro* studies demonstrated that the engineered nanomaterials are able experimentally to cause a wide variety of toxic effects. The toxicity depends on their chemical-physical characteristics and in particular by their chemical composition, the diameter and shape, high area/surface ratio, and the possible state of aggregation/agglomeration (Borm et al., 2006; Nel et al., 2006).

The results of *in vitro* studies showed that different types of nanomaterials are able to induce marked oxidative stress in cell cultures, as demonstrated by the intracellular levels increase of reactive oxygen species (ROS), in oxidation of organic molecules and the increased activity of antioxidant enzyme systems such as glutathione peroxidase (GSH) (Lin et al., 2006).

Instead, several *in vivo* studies on the toxicokinetics of different engineered nanomaterials demonstrated their ability to be absorbed through many ways and reach through the bloodstream or lymphatic system, different organs and tissues, which can lead to adverse health effects (Landsiedel et al., 2012).

It is known that the majority of industrial and urban waste end up in the rivers and coastal waters, because of the extremely small size of the nanoparticles. Release of nanoparticles into the sea raise new doubts that need to be studied in the next future. The potential routes of entry of nanoparticles on aquatic organisms include the direct ingestion, diffusion through the gills and skin (Handy et al., 2008).

Recently, *in vivo* studies performed on *Mytilus galloprovincialis*, bioindicator species used for testing exposure to xenobiotic substances, showed that titanium dioxide nanoparticles (TiO_2_NPs) accumulate in various target organs, especially in gills and digestive gland. The genotoxicity test carried out through Comet Assay revealed a significant dose and time dependent lesion to the DNA (Gornati et al., 2016). Furthermore, TEM analysis showed cellular damages supporting the evidence of an initial inflammatory response by the cells of the target organs leading to apoptosis (Gornati et al., 2016).

The adsorption by the intestinal structures was also demonstrated in rainbow trout (*Oncorhynchus mykiss*) after exposure to TiO_2_NPs both through food (Ramsden et al., 2009) and through the titanium dioxide NPs water dispersion (Federici et al., 2007).

In a previous study (Brundo et al., 2016), the non-toxicity of new synthesized engineered nanomaterials was compared with free Au and TiO_2_ nanoparticles was established by testing the effect of the material on zebrafish larvae using Zebrafish Embryo Toxicity Test (ZFET), an alternative method of animal test (OECD, 2013; Buccheri et al., 2016; Salvaggio et al., 2016). The results obtained showed that neither mortality as well as sublethal effects were induced by the different nanomaterials and nanoparticles tested. Only zebrafish larvae exposed to free gold nanoparticles showed a different response to anti-metallothioneins (MTs) antibody, surely correlated to the dispersion of metal ions in aqueous solution (Brundo et al., 2016).

In this paper, the long term effects of AgNPs in adult specimens of zebrafish was studied. As biomarkers of exposure, we analyzed metallothioneins (MTs). They show to be involved in heavy metal ion homeostasis and detoxification (Ruttkay-Nedecky et al., 2013; Brundo et al., 2016; Pecoraro et al., 2017; Salvaggio et al., 2017). Based on their affinity to metals, in fact, these proteins are able to transport essential metals to place of need or detoxify toxic metals to protect cells. For these reasons the MTs play a key role in the maintaining of metal homeostasis (Ruttkay-Nedecky et al., 2013). The AgNPs concentration found in the treated animals, measured by Inductively Coupled Plasma Mass Spectrometry (ICP-MS).

## Materials and methods

The study was made possible thanks to the collaboration between the Fish Pathology and Experimental Centre of Sicily (CISS) of the Department of Veterinary Science (University of Messina) which has provided zebrafish specimens and the CNR-IMM which has produced silver nanoparticles. The use of 40 adult subjects set up for this trial was approved by the Italian Health Ministry (authorization n°1244/2015-PR).

### Nanoparticles characterization

Synthesis of the nanoparticles is performed by the PLAL (Pulsed Laser Ablation in Liquids) method: a physical process that involves the use of nanosecond laser energy pulses on a substrate immersed in a solvent. The substrate absorbs the laser pulse releasing material which realizes nanoparticles directly in liquid. Scanning Electron Microscopy SEM (Figure 1) and dynamic light scattering (DLS) (not shown here) show that nanoparticles are spherical in shape and 50 nm in diameter. Nanoparticles are negatively charged having a Zeta potential of −40 mV at pH 7. Nanoparticles are stable for several days after preparation.

**Figure 1:** Scanning electron microscope (SEM). SEM image of AgNPs synthetized by pulsed laser ablation in liquid.

SEM images were acquired by using a Field Emission SEM (Gemini Zeiss SUPRA™25) at working distance of 5–6 mm, using an electron beam of 5 KeV and an in-lens detector. DLS and zeta potential measurements are performed with a homemade apparatus described elsewhere (Zimbone et al., 2012) The sample was lighted with a 660 nm diode laser by using a power of 10 mW.

Since the nanoparticles are photosensitive, they were kept in the darkness at the temperature of 4°C until use.

### Silver quantification through ICP-MS analysis

Metal silver extraction performed by microwave digestion (Milestone Ethos 1 FKV, Bergamo, Italy). AgNPs solutions sonicated for 2 h; 0.5 g of each analytical sample weighed with an analytical scale (Mettler A30) into a TFM vessel and mineralized in a microwave system with a digestion solution prepared using 7 ml of 65% nitric acid (HNO_3_) and 2 ml of 35% hydrogen peroxide (H_2_O_2_, J.T. Baker). After mineralization (Microwave power 1,500 W, temperature 200°C), the vessels were opened, the solutions transferred into flasks and ultrapure water (Millipore Merck) was added to the samples up to final volume. A standard Silver ICP (Sigma-Aldrich, Milan, Italy) and the calibration curve used with the method of the standard solution diluted to various concentrations with a range 1–100 ppb (μg/l).

Ag content carried out by Inductively Coupled Plasma Mass Spectrometry (ICP-MS) under following conditions:

- Octapolo ICP-MS Agilent 7500 (Santa Clara, CA, USA) equipped with a Autosampler ASX 500;
- Radio frequency of 1.5 kW;
- Make-up gas at a flow rate of 0.24 l/min;
- Carrier gas at a rate of 0.88 l/min;
- Argon as the plasma gas with a flow rate of 15 l/min.

^45^Sc, ^89^Y, ^182^W were used as internal standard, at a concentration of 100 mg/kg.

The quantitative analysis performed using a calibration curve (R^2^ > 0.997). The detection limit for silver was <1 μg/kg. The SEM analysis conducted on polished graphite plates through the drying of a few drops of AgNPs mother solution after appropriate sonication.

### Fish care

Before starting experimentation, animals used for our studies were housed for a long time in the Fish Facility (Zeb Tech, Stand-Alone). It was provided a constant daily nutrition and natural physical/chemical conditions as photoperiod (14:10 light:dark), temperature (27°C) and pH (7,5) ensuring the highest animal welfare as it established by the World Organisation for Animal Health.

### Experimental phase

We have evaluated the possible toxicity of three increasing concentration of AgNPs (8, 45, and 70 μg/l) for a period of 30 days. NPs concentrations were chosen by the CNR starting from preliminary experiments conducted on nanosystems (Scuderi et al., 2014; Brundo et al., 2016) and from literature data (Muth-Köhne et al., 2013). Three different solutions were prepared daily starting from stock particle solution, added to the standalone facility water and sonicated for 4 cycles. Each cycle was 15 min with 5 min of break using a probe sonicator (FALC Labsonic LBS2) with a frequency of 40 kHz under extractor fan, in order to disrupt any possible aggregates. Zebrafish were randomly selected, mixed between male and female, subdivided in 4 groups (CTRL, NPa, NPb, NPc) each one of them composed of 10 fishes and introduced in 2 l of AgNPs solution. Zebrafish were maintained in tanks equipped with aeration and fed daily. The fish behavior was evaluated visually after 0, 3, 6, and 24 h after exposure to silver nanoparticles in order to reveal a change in swimming speed, loss of balance, respiration and any possible abnormal behavior. Every day, eventual fish mortality was recorded.

### Histopathology

At the end of the experimental period, adult of zebrafish have been carefully euthanized by anesthesia with a dose of 0.7 g/l tricaine methane sulfonate (MS-222) buffered. Gills, liver, gut were excised and immediately fixed in 4% formaldehyde (Bio-Optica) in PBS buffered (Phosphate Buffered Saline, Sigma Life Science) at room temperature for 24 h.

Gills were decalcified, prior to processing, with a decalcifier agent (Biodec R, Bio-Optica) for 2 h at room temperature. Histological examinations were performed according to our standard laboratory procedures. All tissues were washed three times with PBS (0.1 M, pH 7.4), gradually dehydrated in ascending alcohols series (35°, 50°, 70°, 95°, absolute ethanol) for 20 min each one and clarified in xylene for 1 h at room temperature, subsequently embedded in paraffin wax (Medite tissue wax 56–58°C). Five μm thick histological sections cut by microtome (Reichert Jung 1150 Autocut) and collected on glass slides (Menzel Gläser, Thermo Scientific). At least 10 slides of each tissue were collected. The sections were stained with Haematoxylin-Eosin (HE) (Bio-Optica) (Brundo et al., 2011) and observed under optical microscope (Leica DM750) to identify potential morphological alterations. Photographs were produced using an optical microscope (Leica DMLB) equipped with a digital camera (Leica DFC500).

### Immunoistochemistry

The immunohistochemical protocol was performed on the gills, liver and intestine sections to detect MTs proteins using the indirect method of conjugation of an anti-mouse-MT 1 primary antibody (Santa Cruz Biotechnology, CA, USA) diluted 1:1,000 and TRITC-conjugated goat anti-mouse IgG secondary antibody (1:1,000, Sigma-Aldrich). The sections were dewaxed overnight in xylene, rehydrated in descending alcohols series (until tap water) and then were incubated with 1% BSA-PBS buffered in a humid chamber at 4°C for 20 min. It follows incubation with primary antibody at 4°C overnight. After rinsing with PBS, sections incubated in TRITC-conjugated secondary antibody for 1 h at 4°C in darkness. Finally, fast dehydration in increasing alcohol (70°, 80°, 95°) and mounting with antifade mounting medium containing DAPI (Vectashield, Vector Laboratories) were realized. Observations were carried out using a microscope ZEISS AXIO Observer Z1 with Apotome2 system, equipped with the ZEN PRO software.

### Western blotting analysis

The samples were homogenized in a lysis buffer (Tris–HCl 40 mM, EDTA 25 mM, 0.2% SDS, pH 7.4). Total protein concentration was determined according to the Bradford method (Bradford, 1976). Thirty micro gram of protein/lane was analyzed by minigel SDS-PAGE and transferred to a nitrocellulose membrane using Transblot (Biorad). The proteins levels were measured by incubating nitrocellulose membranes overnight at 4°C with mouse monoclonal primary antibody anti-MT 1 (1:1,000, Santa Cruz Biotechnology, CA, USA). The complex protein-primary antibody was detected using a HRP-conjugated Ig-G anti-mouse secondary antibody (1:2,000, Abcam) by chemiluminescent method. Blots were scanned and quantified by a specific software (Image J).

### Gene expression analysis

RNA was extracted by Trizol reagent (Invitrogen, Carlsbad, CA, USA). First strand cDNA was then synthesized with Applied Biosystem (Foster City, CA, USA) reverse transcription reagent. MT 1 mRNA expression was assessed using a fuorescence-based real-time detection method by 7900 HT Fast Real Time PCR System (Life technologies, Carlsbad, CA, USA). For each sample, the relative expression level of MT 1 mRNA (forward primer 5′-GCC AAG ACT GGA ACT TGC AAC-3′; reverse primer 5′-CGC AGC CAG AGG CAC ACT-3′; amplicon size is 130 bp) was normalized using β-actin 2 (forward primer 5′-CTT GGG TAT GGA ATC TTG CG-3′; reverse primer 5′-AGC ATT TGC GGT GGA CGA T-3′; amplicon size is 88 bp) as an invariant control. The relative mRNA expression level was calculated by the threshold cycle (Ct) value of each PCR product and normalized with that of β-actin 2 by using comparative 2^−ΔΔ^Ct method.

### Statistical analysis

Statistical analysis was made with Prism Software (Graphpad Software Inc., La Jolla, CA, USA). Data were expressed as mean or SD. Statistical analysis was carried out by two-way ANOVA test. A *p*-value of 0.05 was considered to indicate a statistically significant difference between experimental and control groups.

## Results and discussion

Histological observation of tissues at the end of the experiment showed normal anatomy in the freshwater controls. Gills structure, both primary and secondary lamellae, appeared intact and well recognizable as well as chloride cells, pillar cells and mucosal ones too (Figure 2A). A whole intestinal lumen and well lying microvilli appeared in the gut histological sections (Figure 3). On the contrary, silver nanoparticles caused damage to the gills structure such as sub-epithelial edema, hyperplasia (Figures 2B,C), lamellar fusion (Figure 2B), as well as teleangectasia (Figure 2D). The necrosis of intestinal villi with reduction of their length was also demonstrated in the gut (Figures 3B–D).

**Figure 2:** Gills morphology images. **(A)** CTRL: gills structure, both primary and secondary lamellae, appeared intact and well recognizable as well as chloride cells, pillar cells and mucosal ones too. **(B–D)** gills structure after 30 days to exposure AgNPs: **(B)** NPa; **(C)** NPb; **(D)** NPc. Exposure to silver nanoparticles caused damage to the gills structure such as sub-epithelial edema, hyperplasia **(B,C)**, lamellar fusion **(B)**, as well as teleangectasia **(D)**. Scale barr: **A** = 120 μm; **B,D** = 80 μm; **C** = 40 μm.

**Figure 3:** Gut morphology images. **(A)** CTRL: A whole intestinal lumen and well lying microvilli appeared in the gut histological sections. **(B–D)** Gut structure after 30 days to exposure AgNPs: **(B)** NPa; **(C)** NPb; **(D)** NPc. Exposure to silver nanoparticles caused necrosis of intestinal villi with reduction of their length was also demonstrated in the gut **(B–D)**. Scale barr: **A** = 250 μm; **B,D** = 200 μm; **C** = 50 μm.

No alterations have observed in liver tissue as shown in Figure 4. In this image, a clear distinction can be made between the male and female liver in the adult zebrafish. The female hepatocytes are very basophilic as a result of the production of vitellogenin (Menke et al., 2011).

**Figure 4:** Liver morphology images. Liver structure after 30 days of exposure to 70 μg/l AgNPs no showed never cytological alterations: **(A)** female; **(B)** male. Scale barr: A and B = 100 μm.

However, dose dependent effects of nanosilver suspensions with significantly greater damage were observed at lower concentrations.

The immunohistochemical examination highlighted the presence of metallothioneins. Metallothioneins are substrates inducible proteins in the presence of metal ions and show a very high affinity toward them. Several studies support the use of MTs. Copat et al. (2012) have shown that MTs are a potential biomarker for contamination in the aquatic environment metals; Brundo et al. (2016) found that zebrafish embryos exposed to gold nanoparticles showed a positive response to anti-MT 1, pointing out that the metal nanoparticles can promote synthesis of inducible MTs.

The slight positivity of MTs found in the control group is a normal physiological condition because these organs represents one of the first sites of defense against xenobiotics.

Using specific antibodies anti-MT 1, it has been showed a clear expression of these proteins in the intestinal tissues AgNPs treated (Figures 5B,C), compared with the control group (Figure 5A). The same results were obtained for the liver and the gills (Figure 6). The WB analysis did not show any difference in the expression of MT1 in each tested concentration, but only differences tissue-dependent (Figure 7).

**Figure 5:** MT 1 expression in gut tissue. Using specific antibodies anti-MT, it has been showed a clear expression of these proteins in the intestinal tissues AgNPs treated compared with the control group. **(A)** CTRL; **(B)** NPa; **(C)** NPc. Scale barr: **A–C** = 200 μm.

**Figure 6:** MTs expression in liver **(A)** and gills **(B)** tissue. Liver and gills structure after 30 days of exposure to 70 μg/l AgNPs showed a clear expression of metallothioneins. Scale barr: **A,B** = 10 μm.

**Figure 7:** Western blotting analysis. The MT1 level in zebrafish after exposure to 70 μg/l Ag free nanoparticles. The data are expressed as mean + SEM. Statistical analysis was carried out by ANOVA test. A *p*-value of less than 0.05 (*p* < 0.05) was accepted as statistically significant.

It was also observed a higher response at lower concentration of mt 1 mRNA expression, in all three tissue treated (Figure 8).

**Figure 8:** mRNA gene expression of MT1 in zebrafish after exposure to Ag free nanoparticles. Bars represent the mean ± SEM of three independent experiments. Statistical analysis was carried out by ANOVA test. A *p*-value of less than 0.05 (*p* < 0.05) was accepted as statistically significant between experimental and control groups. (Calculated value of 2^−ΔΔCt^ in untreated sample was 1).

Results obtained through the different applied methods showed that silver nanoparticles have caused tissue damage because they were absorbed in the body.

Assuming a purely preliminary conceptual analysis, we would expect a corresponding increase of the lesions correlated to the growing nanoparticles concentration both in gill and gut tissues.

Instead, the group of zebrafish exposed to the highest concentration had a lower degree of toxicity compared to the group treated with NPs lower concentrations. These results suggested that as high is the concentration as high is the probability that the particles aggregate, and little by little their size increase, the absorption capacity of the exposed tissues may reduce. Instead, in the solution with the lower concentration of NPs, silver nanoparticles are mono-dispersed and more easily adsorbed by gills and intestine.

The ICP-MS analysis infact shows that the amount of particles absorbed in all treated samples is almost the same. Total silver concentrations found vary from a minimum of 6 mg/l in NPa group samples to 8.2 mg/l in those belong to NPc group. The rate of absorption was respectively of 76.1% (NPa), 14.5% (NPb) and 11.7% (NPc), demonstrating a greater capacity of assimilation of the particles in mono-dispersed phase (Figure 9).

**Figure 9:** Graphic results of ICP-MS analysis. The ICP-MS analysis infact shows that the amount of particles absorbed in all treated samples is almost the same. Total silver concentrations found vary from a minimum of 6 mg/l in NPa group samples to 8.2 mg/l in those belong to NPc group. The rate of absorption was respectively of 76.1% (NPa), 14.5% (NPb), and 11.7% (NPc), demonstrating a greater capacity of assimilation of the particles in mono-dispersed phase.

For this reason, it is possible affirm that the toxicity of silver nanoparticles is related to their size and degree of dispersion rather than their concentration.

Therefore, it is necessary that the NPs solutions undergo sonication during the whole period of the trial in order to prevent the possibility of aggregation and make them more bioavailable for animals used for ecotoxicological tests.

These results suggest that AgNPs can generate different degrees of toxicity. The bioavailability of silver nanoparticles, in fact, is an important parameter of toxicity to aquatic organisms and depends on many factors such as sedimentation, aggregation and particle size.

## Conclusion

It is important to consider that the design of nanoparticles comparable in size to biological molecules allow their easy incorporation into biological systems causing modification. Based upon size alone, nanoparticles can exploit the host circulatory system for transport in the body and enter, translocate, and damage living tissues by penetrating physiological barriers. In this study, we have demonstrated that silver nanoparticles dispersed in water are able to cross the mucosal barriers, producing a damage that goes to the detriment of these districts. The damn to the mucosal epithelium of the gills, and to a lesser degree to the intestinal tissue, is however reversible, because no damage of the basal membrane was ever demonstrated.

The purpose of this study was to assess the chronic effects of silver nanoparticles on aquatic organisms. Having proved that AgNPs cause damages to the tissues, we hope for this study is a useful contribution for scientific community to establish other environmental regulations. Furthermore, it would be appropriate to make further examinations for the marine waters by the authority, especially for the coastal waters, and possibly, establish new limits of the law in order to protect human health as well as animal species and the environment after further investigations on nanoparticles toxicity.

Silver nanoparticles are used in various applications; in the medical and aquaculture fields they are employed for their well-known antimicrobial abilities. In the aquaculture, the use of nanoparticles is still under study targeted mainly to water treatment depuration and defense against pathogens. Nanotechnologies can be useful to solve most of the problems in aquaculture but their use should be taken with care to avoid polluting the environment.

## Author contributions

MVB, RP, and FM have carried out the planning of experiments, have elaborated the data and have drafted the manuscript; FC, GD, and CI have carried out experiments on zebrafish and hystological analysis; RP, EMS, and DT have carried out experiments of western blotting, immunohistochemical analysis and gene expression analysis; AntS and GG have revised the manuscript; AndS and AR have carried out ICP_MS analysis; MZ and GI have realized NPs and have revised the manuscript.

### Conflict of interest statement

The authors declare that the research was conducted in the absence of any commercial or financial relationships that could be construed as a potential conflict of interest.
